# An Ensemble of Deep Learning Enabled Brain Stroke Classification Model in Magnetic Resonance Images

**DOI:** 10.1155/2022/7815434

**Published:** 2022-11-18

**Authors:** Ala' A. Eshmawi, Mashael Khayyat, Abeer D. Algarni, Inès Hilali-Jaghdam

**Affiliations:** ^1^University of Jeddah, College of Computer Science and Engineering, Department of Cybersecurity, Jeddah, Saudi Arabia; ^2^University of Jeddah, College of Computer Science and Engineering, Department of Information Systems and Technology, Jeddah, Saudi Arabia; ^3^Department of Information Technology, College of Computer and Information Sciences, Princess Nourah Bint Abdulrahman University, P.O.Box 84428, Riyadh 11671, Saudi Arabia; ^4^Department of Computer Science and IT, College of Community, Princess Nourah Bint Abdulrahman University, P.O.Box 84428, Riyadh 11671, Saudi Arabia

## Abstract

Brain stroke is a major cause of global death and it necessitates earlier identification process to reduce the mortality rate. Magnetic resonance imaging (MRI) techniques is a commonly available imaging modality used to diagnose brain stroke. Presently, machine learning (ML) and deep learning (DL) models can be extremely utilized for disease detection and classification processes. Amongst the available approaches, the convolutional neural network (CNN) models have been widely used for computer vision and image processing issues such as ImageNet, facial detection, and digit classification. In this article, a novel computer aided diagnosis (CAD) based brain stroke detection and classification (CAD-BSDC) model has been developed for MRI images. The proposed CAD-BSDC technique aims in classifying the provided MR brain image as normal or abnormal. The CAD-BSDC technique involves different subprocesses such as preprocessing, feature extraction, and classification. Firstly, the input image undergoes preprocessing using adaptive thresholding (AT) technique for improving the image quality. Followed by, an ensemble of feature extractors such as MobileNet, CapsuleNet, and EfficientNet models are used. Besides, the hyperparameter tuning of the deep learning models takes place using the improved dragonfly optimization (IDFO) algorithm. Moreover, satin bowerbird optimization (SBO) based stacked autoencoder (SAE) is used for the classification of brain stroke. The design of optimal SAE using the SBO algorithm shows the novelty of the work. The performance of the presented technique was validated utilizing benchmark dataset which includes T2-weighted MR brain image collected from the axial axis with size of 256 × 256. The simulation outcomes indicated the promising efficiency of the proposed CAD-BSDC technique over the latest state of art approaches in terms of various performance measures.

## 1. Introduction

Strokes are the 3rd most common cause of death around the world as per the report of the world health organization (WHO). With around 87% the more common type are ischemic strokes, caused by disturbance in the brain blood supply. Measuring volume and lesion location could assist diagnoses and guide treatment decisions [1]. Moreover, lesion classification plays a significant role in cognitive neuroscience research. This frequently includes an anatomical analysis, where brain area is associated with the neurological deficit that requires manual examinations of massive stroke image databases. Hence, an automated methodology for segmenting ischemic lesions in brain images is extremely needed [2, 3]. Ischemic stroke lesions undergo several developmental stages. The moment of partial or total loss of blood supply to the infected brain areas is called the onset of the stroke and marks the beginning of the hyperacute stage. At onset, the infection areas are separated into a core of infarcted tissue and a surrounding penumbra of under perfused, however possibly salvageable tissue i.e., partially provided by collateral blood flow [4]. The stroke developmental phase is related to amount of cell death and reconstructing mechanism which affects visibility of the stroke area in magnetic resonance imaging (MRI), mostly by the migration of water molecules [5].

Brain imaging methodologies, namely, computed tomography (CT) and MRI are very supportive for a physician for starting the early screening of the patients [6]. Also, there are several imaging modalities for analyzing brain that might involve diffuse optical imaging, X-ray imaging, positron emission tomography, magnetoencephalography, and functional MRI [7]. But this imaging technique requires well-trained operators and higher operating costs, thus many of these imaging methods may not be presented in every hospital and clinic. Image classification is broadly utilized in medical imaging systems [8]. But the classification method outcomes must be closer to the manual diagnoses.

This study introduces a novel computer aided diagnosis (CAD) based brain stroke detection and classification (CAD-BSDC) model on MRI images. The proposed CAD-BSDC technique involves preprocessing using adaptive thresholding (AT) technique to improve the image quality. In addition, an ensemble of feature extractors such as MobileNet, CapsuleNet, and EfficientNet models are used. Besides, the hyperparameter tuning of the deep learning models takes place using the improved dragonfly optimization (IDFO) algorithm. Furthermore, satin bowerbird optimization (SBO) based stacked autoencoder (SAE) is used to classify the MR brain image as normal or abnormal. The experimental result analysis of the CAD-BSDC technique takes place utilizing benchmark dataset which comprises T2-weighted MR brain images.

## 2. Literature Review

Currently, deep learning (DL) method was widely utilized as a classification system since it calculates features automatically within the convolution layer of the deep system [9]. The major benefit of utilizing DL method is that it outperforms other traditional methodologies for the classification of images. Several DL methodologies have existed like deep belief nets (DBN), RNNs, LSTM, and so on. Amongst this method, convolutional neural network (CNN) was widely employed in medical image processing and computer vision challenges such as house numbers digit classification, ImageNet, patch classification from medical images, face recognition, and so on [10].

Nishio et al. [11] evaluated and developed an automated acute ischemic stroke (AIS) detection method including 2-phase DL models. Next, the 2-phase method implemented the AIS recognition system in the testing set. To evaluate the detection outcomes, a board-certified radiologist assessed the testing set head CT image with and without help of detection system [12]. Hilbert et al. [13] examined DL methods to build model to directly forecast better reperfusion afterward endovascular treatment (EVT) and better functional outcomes using CT images. This model does not need image annotation and is faster to calculate. The study compared DL to ML methods using conventional radiological image biomarkers. Pan et al. [14] investigated a new method based mainly on DL-ResNet for detecting infarct cores on non-contrast CT images and enhancing the performance of acute ischemic stroke diagnoses. They endlessly enrolled magnetic resonance diffusion weighted image (MR-DWI) confirmed first-episode ischemic stroke patients. Next, utilize decision curve analysis (DCA) model for analyzing the values of this technique in medical settings.

Zhang et al. [15] introduced a DL method that leverages MRI diffusion series for classifying TSS based medically validated threshold. Also, the study presented an intradomain task-adoptive transfer learning technique that includes model training on simple medical tasks (stroke recognition) and refined the method with distinct binary thresholds of TSS. Wang et al. [16] evaluated and developed a DL based method to assist the selection of appropriate patients with acute ischemic stroke for endovascular treatment-based 3D pseudo-continuous arterial spin labeling (pCASL). The DL and six ML methods have been trained by using 10-fold CV.

## 3. The Proposed Model

In this study, a new CAD-BSDC model has been developed for MRI images for classifying them into normal or abnormal. The CAD-BSDC technique involves different subprocesses such as AT based preprocessing, ensemble of feature extraction, IDFO-based hyperparameter tuning, SAE-based classification, and SBO-based parameter tuning.  Figure 1 illustrates the overall process of CAD-BSDC technique.

### 3.1. Image Preprocessing Using at Technique

At the primary level, the AT technique is applied on MRI images to remove the noise and enhance the quality. It is an effective method to determine the infected regions by the use of thresholding concept. In the AT technique, the investigation of the MRI images takes place for the distributed pixel intensities and the threshold value is chosen. In this case, the input MRI image can be denoted as *g*(*x*, *y*), *I* implies the threshold value, and the final image can be defined as *f*(*x*, *y*). It can be mathematically defined as follows [17]:

(1) $$\begin{array}{c} f\left(x,y\right)=\left\{\begin{array}{cc} 1, & g\left(x,y\right)\geq I,\\ 0, & \text{otherwise}. \end{array}\right\} \end{array}$$

### 3.2. Ensemble of Feature Extraction Approaches

During the feature extraction process, the ensemble of feature extractors namely MobileNet, CapsuleNet, and EfficientNet models are used. The DL is a type of CNN and has extremely utilized for images [18]. In recent times, DL was extremely utilized in the analysis of several medicinal diseases. Also, several researchers are developed by analysis of skin disease utilizing DL. The DL has several linked layers using distinct weight as well as activation functions. A fundamental DL technique involves convolution, pooling, and connected layers. Many activation functions were utilized for adjusting the weight. During this case, EfficientNetB3 was utilized for glaucoma detection. The EfficientNetB3 is current, cost-efficient, and robust technique established by scaling 3 parameters namely depth, width, and resolution [19]. An EfficientNetB3 method with noisy-student weight was utilized from scenarios I and III to the transfer learning (TL) procedure, but “isicall_eff3_weights” weight is utilized as pretrained to scenarios II and IV. The GlobalAveragePooling2D layers were added to all scenarios for generalizing the optimum model. The amount of parameters is decreased. Also, the rectified linear unit (ReLU) activation function was utilized with 3 dense and 2 dropout layers. The resultant layer has several outcome units to multiclass classification utilizing the softmax activation functions.  Figure 2 demonstrates the structure of CapsNet.

The MobileNet [20] has lesser framework, minimum computation, and superior precision that is utilized to mobile terminal and embedding devices. According to depthwise separable convolutional, MobileNets utilize 2 global hyperparameters for keeping a balance amongst efficacy and accuracy. The basic concept of MobileNet is decomposition of convolutional kernel. With utilizing depthwise separable convolutional, the typical convolutional was decomposed as to depthwise convolutional and pointwise convolutional with convolutional kernels. The depthwise convolutional filter execute convolutional for all channels, and convolutional was utilized for combining the outcomes of depthwise convolutional layer. During this technique, *N* typical convolutional kernel. The typical convolution filters integrate an input as to a novel group of outputs, but the depthwise separable convolutional separates the inputs as to 2 layers, one to filter and another to merge. The MobileNetV2 establishes novel components with inverted remaining framework.

In order to compensate for shortcomings of CNN, the network framework named the CapsNet was presented [21]. The CapsNet is a deep network technique involving capsules. The capsule was comprised of a set of neurons. The activation neuron signifies the features of modules from the objects. All the capsules are responsible to determine a single module from the object, and every capsule jointly defines the entire framework of objects. Conversely, for any DNNs (for instance, DBN), this framework preserves object modules and spatial data. Related to CNN, the CapsNet was comprised of multi-layer networks.

### 3.3. Hyperparameter Tuning Using IDFO Algorithm

For optimally adjusting the hyperparameters of the DL models, the IDFO algorithm is applied. The DFO method was coined by Mirjalili at Griffith University in 2016 [22]. This method is a meta-heuristic approach-based SI is stimulated by dynamic as well as static behaviors of dragonflies in nature. There are 2 primary phases of optimization: exploitation and exploration. These two stages are modelled by dragonflies, either statically or dynamically searching for food or avoiding the enemy. The 2 further behaviors are added to these three fundamental behavior in *DA*: move to the food and avoid the enemy. Thus, once each individual moves to food source (equation (5)), they need to avoid the enemy simultaneously (equation (6)).

(2) $$\begin{array}{c} S_{i}=-\sum_{j=1}^{N}X-X_{j},\\ A_{i}=\frac{\overset{N}{\underset{j=1}{\sum }}V_{j}}{N},\\ C_{i}=\frac{\overset{N}{\underset{j=1}{\sum }}X_{j}}{N}-X,\\ F_{i}=X^{+}-X,\\ E_{i}=X^{-}+X, \end{array}$$

where, *X* indicates the immediate location of the individual, in which *X*_*j*_ indicates the immediate location of *j*^*th*^ individual. *N* characterizes the amount of neighboring individuals, in which *y*_*j*_ shows the speed of *j*^*th*^ neighboring individual. *X*^+^ and *X*^−^ denotes the position of the food and enemy source, correspondingly [23]. The overall steps of the DFO algorithm are given in 1.

To upgrade the place of artificial dragonflies in the searching space and simulate the motion, two vectors are taken into consideration: position (*X*) and step (*X*). The step vector considers as speed, shows the direction of dragonfly motion (equation (7)). Then estimating the step vectors, the position vector is upgraded (equation (8)):

(3) $$\begin{array}{c} \nabla X_{t+1}=\left(sS_{i}+aA_{i}+cC_{i}+fF_{i}+eE_{i}\right)+w\nabla X_{t},\\ X_{t+1}=X_{t}+\nabla X_{t+1}. \end{array}$$

In which, and *f*, *e*, *w*, and *t* represents the food factor, enemy factor, inertia coefficient, iteration number, correspondingly and the, *a*, and *c* indicates separation, alignment, and cohesion coefficient, correspondingly. This coefficient and the abovementioned factor enable to implementation of exploitative and exploratory behaviors. In the IDFO algorithm, the traditional DFO algorithm is integrated into the flower authorization algorithm, we set the value ranges [*S*_min_,  *S*_max_]. To efficiently evade the situation where the dragonfly collectively gathers in the first phase, the uniform distribution is utilized for implementing random initialization process on all the dimensions [24],

(4) $$\begin{array}{c} x_{\text{id}}^{0}=S_{\text{min}}+\left(S_{\text{max}}-S_{\text{min}}\right). \end{array}$$

Afterward preprocessing, the 2 procedures are further merged for guiding the dragonfly to fly to an optimal location.

### 3.4. Image Classification Using SBO-SAE Model

Finally, the SBO-SAE model can be employed for the classification of MRI images. The SAE is developed based on the concept of auto encoder (AE). In SAE model, the encoding part of the AE is stacked together, i.e., the input of initial layer of an AE model is actual data and the input of lower layer is hidden layer data. Lastly, a classification model is appended to the network [25]. The training process of the SAE model involves the pretraining and the inverse fine-tuning procedure. It makes use of a huge quantity of unlabeled data for unsupervised learning, independently extracted the features, and utilizes the labelled data for inverse fine tuning of the network. For boosting the performance of the SAE technique, the weight and bias values are optimally chosen by the SBO algorithm.

SBO technique begins generating a primary uniform arbitrary population that contains a group of places to bower [26]. All positions (pop(i).Pos) are determined to the parameter which is supposed that optimize as written in equation (6). It could be noticeable the value of primary population lie among the existing minimal as well as maximal limit of optimizing parameters.

(5) $$\begin{array}{c} \text{pop }\left(i\right)\;\cdot Pos\;=\text{rand}\left(1,\;n_{\text{var}}\right)\cdot \left({\text{Var}}_{\text{Max}}-{\text{Var}}_{\text{Min }}\right)+{\text{Var}}_{\text{ Min }},\;\forall i\in n_{\text{Pop}}. \end{array}$$

Comparatively, same as ABC, the probability of fascinating of male/female (Prob_*i*_) to bower was calculated as follows.

(6) $$\begin{array}{c} {\text{Prob}}_{i}=\frac{\text{cos}t_{i}}{\sum_{k=1}^{n_{\text{Pop}}}\text{cos}t_{i}},\;\forall i\in n_{\text{Pop}},\\ \text{cos }t_{i}=\left\{\begin{array}{cc} \frac{1}{1+f\left(x_{i}\right)}, & f\left(x_{i}\right)\geq 0,\\ 1+\left|f\left(x_{i}\right)\right|, & f\left(x_{i}\right)<0. \end{array}\right) \end{array}$$

Same as other evolutionary dependent upon optimizer, elitism was utilized for storing an optimum solution(s) at all iterations of optimized procedure. In the mating season, males like every other bird utilize its drives for building and decorating the bower. Noticeably, older and experienced males are appealed further attention of others to their bower. Conversely, this bower has further fitness than the other bower. During the SBO processes, the place of an optimum bower created by bird was estimated as elite of *k*^*th*^ iteration (*x*_elite,*k*_) that is maximum fitness and is capable of affecting the other places. In all iterations, a novel modification at some bower was computed dependent upon equation demonstrated in

(7) $$\begin{array}{c} \chi_{ik}^{\text{new}}=\chi_{i,k}^{\text{old}}+\beta_{k}\left[\left(\frac{x_{jk}+x_{\text{elite},k}}{2}\right)-\chi_{i,\;k}^{\text{old}}\right]. \end{array}$$

It can be worth maintaining that roulette wheel selective process was utilized for picking up bower with superior probability (*x*_*jk*_). In SBO, Parameter *β*_*k*_ defines the count of steps for selecting target bowers that are calculated to all variables and modified based on

(8) $$\begin{array}{c} \beta_{k}=\frac{\alpha }{1+{\text{Prop}}_{i}}. \end{array}$$

Arbitrary modifies were executed to *x*_*ik*_ with specific probability, where normal distribution (N) has been utilized with average of *x*_*i*,*k*_^old^ and variance of *σ* as stated in equation.

(9) $$\begin{array}{c} X_{ik}^{\text{ne}\omega }∼X_{ik}^{\text{old}}+\sigma \cdot N\left(0,1\right),\\ \sigma =Z\cdot \left({\text{Var}}_{\text{Max}}-{\text{Var}}_{\text{Min}}\right). \end{array}$$

Finally, all the cycle is an old population and population attained in modifies as aforementioned were evaluated, integrated, sorted and novel population was created. The pseudocode of SBO algorithm is given in 2.

The SBO approach develops a FF for attaining enhanced classification efficiency. It defines a positive integer for representing the optimum efficiency of candidate solution. During this case, the minimized classification error rate was regarded as FF is provided in equation (10). The optimum solutions have reduced error rates and the worst solutions obtain an enhanced error rate.

(10) $$\begin{array}{c} \text{fitness}\left(x_{i}\right)=\text{ClassifierErrorRate}\left(x_{i}\right),\\ =\frac{\text{number of misclassified instances}}{\text{total number of instances}}*100. \end{array}$$

## 4. Experimental Validation

The performance validation of the CAD-BSDC technique takes place using the benchmark dataset [27], which contains MRI images under six distinct classes. The details relevant to the dataset are given in Table 1.  Figure 3 shows the sample MRI images.

Figure 4 shows the confusion matrices offered by the CAD-BSDC technique on the classification of brain stroke. The figure shows that the CAD-BSDC technique has effectually identified distinct classes of brain stroke. For instance, under 500 epochs, the CAD-BSDC technique has categorized 23 images in class 0, 24 images under class 1, 24 images in class 2, 52 images under class 3, 24 images in class 4, and 22 images in class 5, respectively. Simultaneously, in 1000 epochs, the CAD-BSDC approach has classified 23 images under class 0, 22 images in class 1, 24 images in class 2, 54 images under class 3, 23 images in class 4, and 22 images in class 5 correspondingly. Furthermore, under 1500 epochs, the CAD-BSDC methodology has classified 25 images in class 0, 21 images under class 1, 22 images in class 2, 52 images in class 3, 26 images in class 4, and 23 images in class 5 correspondingly. Furthermore, under 2000 epochs, the CAD-BSDC system has categorized 25 images in class 0, 20 images in class 1, 23 images in class 2, 54 images under class 3, 26 images in class 4, and 23 images in class 5 correspondingly.

Table 2 offers a detailed classification result analysis of the CAD-BSDC technique under various classes and epoch counts. The results ensured the effective performance of the CAD-BSDC technique interms of different measures.

Table 3and Figure 5 depict the overall classification result analysis of the CAD-BSDC technique under varying epochs. The results show that the CAD-BSDC technique has resulted in improved classification results. For instance, with 500 epochs, the CAD-BSDC technique has resulted in the *sens*_*y*_, *spec*_*y*_, *accu*_*y*_, *prec*_*n*_, *F*_score_, and MCC of 94.71%, 99%, 98.31%, 94.63%, 94.55%, and 93.61%, respectively. As well as, with 1000 epochs, the CAD-BSDC process has resulted in *sens*_*y*_, *spec*_*y*_, *accu*_*y*_, *prec*_*n*_, *F*_*score*_,   and MCC of 93.35%, 98.83%, 98.13%, 94.55%, 93.82%, and 92.78% correspondingly. Furthermore, with 1500 epochs, the CAD-BSDC method has resulted to the *sens*_*y*_, *spec*_*y*_, *accu*_*y*_, *prec*_*n*_, *F*_score_, and MCC of 94.63%, 99%, 98.31%, 94.71%, 94.44%, and 93.58% correspondingly. Finally, with 2000 epochs, the CAD-BSDC approach has resulted in the *sens*_*y*_, *spec*_*y*_, *accu*_*y*_, *prec*_*n*_, *F*_score_, and MCC of 95.28%, 99.16%, 98.69%, 96.76%, 95.75%, and 95.13% correspondingly.

In order to ensure the improvements of the CAD-BSDC technique, a comprehensive comparison study is made in Table 4 [28].

Figure 6 investigates the comparative accuracy analysis of the CAD-BSDC with recent methods on the test dataset. The figure demonstrated that the FODPSO-SVM technique has accomplished ineffectual outcomes with the least values of accuracy. In line with, the SURF-DT and FODPSO-RF techniques have obtained slightly increased values of accuracy. Followed by, the EM-PSORF and EM-PSOSVM techniques have reached moderately improved accuracy values. Though the SIFT-DT technique has reached near optimal accuracy of 97.25%, the CAD-BSDC technique has accomplished maximum accuracy of 98.36%.

Figure 7 explores the comparative *sens*_*y*_, *spec*_*y*_, and *F*_measure_ analysis of the CAD-BSDC with current methodologies on the test dataset. The figure illustrates that the FODPSO-SVM approach has achieved ineffectual outcomes with the least values of *sens*_*y*_, *spec*_*y*_, and *F*_measure_. In line with, the SURF-DT and FODPSO-RF methodologies have attained slightly improved values of *sens*_*y*_, *spec*_*y*_, and *F*_measure_. Then, the EM-PSORF and EM-PSOSVM algorithms have reached better *sens*_*y*_, *spec*_*y*_, and *F*_measure_ values. Although the SIFT-DT model has reached to near optimum *sens*_*y*_, *spec*_*y*_, and *F*_measure_ of 91.04% 98.23%, and 91.91%, the CAD-BSDC model has attained maximal *sens*_*y*_, *spec*_*y*_, and *F*_measure_ of 94.49%, 99%, and 96.64%.

The above mentioned tables and figures demonstrated that the CAD-BSDC technique has showcased superior performance over the other techniques.

## 5. Conclusion

In this study, a new CAD-BSDC model has been developed for MRI images for classifying them into normal or abnormal. The CAD-BSDC technique involves different subprocesses such as AT based preprocessing, ensemble of feature extraction, IDFO-based hyperparameter tuning, SAE based classification, and SBO based parameter tuning. The experimental result analysis of the CAD-BSDC technique takes place utilizing benchmark dataset which includes T2-weighted MR brain images. The simulation outcomes indicated the promising efficiency of the proposed CAD-BSDC technique over the latest state of art approaches in terms of various performance measures. Thus, the CAD-BSDC technique can be realized in a real time environment to aid physicians. As a part of future extension, the classification performance of the CAD-BSDC technique can be enhanced by the use of DL-based segmentation approaches.

## Figures and Tables

**Figure 1:** Overall process of CAD-BSDC technique.

**Figure 2:** Structure of CapsNet.

**Figure 3:** Sample test images.

**Figure 4:** Confusion matrix of CAD-BSDC technique.

**Figure 5:** Overall classification result analysis of CAD-BSDC technique.

**Figure 6:** Accuracy analysis of CAD-BSDC technique with existing approaches.

**Figure 7:** Comparative analysis of CAD-BSDC technique with existing methods.

**Algorithm 1:** Pseudocode of DFO Algorithm.

**Algorithm 2:** Pseudocode of SBO Algorithm.

**Table 1:** Dataset descriptions.

Categories of MR brain stroke images	Class labels	Dimensions	Number of images
Acute (speech arrest)	Class 0	256 *∗* 256	25
Cerebral haemorrhages	Class 1	256 *∗* 256	25
Fatal stroke	Class 2	256 *∗* 256	24
Normal images	Class 3	256 *∗* 256	54
Subacute stroke (hesitating speech)	Class 4	256 *∗* 256	26
Subacute stroke (loss of sensation)	Class 5	256 *∗* 256	24

**Table 2:** Result analysis of CAD-BSDC technique with different classes and epoch counts.

Classes	Sensitivity	Specificity	Accuracy	Precision	F-score	MCC
Epoch-500						
Class 0	92.00	98.04	97.19	88.46	90.20	88.58
Class 1	96.00	98.69	98.31	92.31	94.12	93.16
Class 2	100.00	98.05	98.31	88.89	94.12	93.36
Class 3	96.30	99.19	98.31	98.11	97.20	96.00
Class 4	92.31	100.00	98.88	100.00	96.00	95.45
Class 5	91.67	100.00	98.88	100.00	95.65	95.13
Average	94.71	99.00	98.31	94.63	94.55	93.61
Epoch-1000						
Class 0	92.00	100.00	98.88	100.00	95.83	95.30
Class 1	88.00	98.69	97.19	91.67	89.80	88.19
Class 2	100.00	98.05	98.31	88.89	94.12	93.36
Class 3	100.00	97.58	98.31	94.74	97.30	96.15
Class 4	88.46	98.68	97.19	92.00	90.20	88.58
Class 5	91.67	100.00	98.88	100.00	95.65	95.13
Average	93.35	98.83	98.13	94.55	93.82	92.78
Epoch-1500						
Class 0	100.00	98.04	98.31	89.29	94.34	93.56
Class 1	84.00	100.00	97.75	100.00	91.30	90.48
Class 2	91.67	99.35	98.31	95.65	93.62	92.67
Class 3	96.30	99.19	98.31	98.11	97.20	96.00
Class 4	100.00	100.00	100.00	100.00	100.00	100.00
Class 5	95.83	97.40	97.19	85.19	90.20	88.77
Average	94.63	99.00	98.31	94.71	94.44	93.58
Epoch-2000						
Class 0	100.00	99.35	99.44	96.15	98.04	97.74
Class 1	80.00	100.00	97.19	100.00	88.89	88.02
Class 2	95.83	100.00	99.44	100.00	97.87	97.58
Class 3	100.00	97.58	98.31	94.74	97.30	96.15
Class 4	100.00	98.03	98.31	89.66	94.55	93.75
Class 5	95.83	100.00	99.44	100.00	97.87	97.58
Average	95.28	99.16	98.69	96.76	95.75	95.13

**Table 3:** Overall Classification result analysis of CAD-BSDC technique.

No. of epochs	Sensitivity	Specificity	Accuracy	Precision	F-score	MCC
Epoch-500	94.71	99.00	98.31	94.63	94.55	93.61
Epoch-1000	93.35	98.83	98.13	94.55	93.82	92.78
Epoch-1500	94.63	99.00	98.31	94.71	94.44	93.58
Epoch-2000	95.28	99.16	98.69	96.76	95.75	95.13
Average	94.49	99.00	98.36	95.16	94.64	93.78

**Table 4:** Comparative analysis of CAD-BSDC technique with existing approaches.

Methods	Sensitivity	Specificity	F-measure	Accuracy
CAD-BSDC	94.49	99.00	96.64	98.36
SIFT-DT model	91.04	98.23	91.91	97.25
SURF-DT model	78.10	95.11	80.15	92.62
EM-PSORF	92.50	95.80	95.17	93.40
EM-PSOSVM	90.40	94.60	93.44	93.20
FODPSO-RF	89.40	93.70	93.54	92.40
FODPSO-SVM	88.30	92.60	91.69	91.70

## Data Availability

Data sharing not applicable to this article as no datasets were generated during the current study.
